This article has been retracted.

# Nursing Care Systematization with Case-Based Reasoning and Artificial Intelligence

**DOI:** 10.1155/2022/1959371

**Published:** 2022-03-09

**Authors:** Malik Bader Alazzam, Nahla Tayyib, Samar Zuhair Alshawwa, Md. Kawser Ahmed

**Affiliations:** ^1^Information Technology College, Ajloun National University, Ajloun, Jordan; ^2^Faculty of Nursing, Umm Al-Qura University, Makkah, Saudi Arabia; ^3^Department of Pharmaceutical Sciences, College of Pharmacy, Princess Nourah bint Abdulrahman University, P.O. Box 84428, Riyadh 11671, Saudi Arabia; ^4^Department of English and Modern Languages, IUBAT- International University of Business Agriculture and Technology, Dhaka, Bangladesh

## Abstract

Of the most popular applications of artificial intelligence (AI), those used in the health sector are the ones that represent the largest proportion, in terms of use and expectation. An investigative systematization model is proposed in the scientific training of nursing professionals, by articulating epistemological positions from previous studies on the subject. In order to validate the model proposed, a prototype was created to present an application that could help nurses in their clinical processes, storing their experiences in a case base for future research. The prototype consisted of digitizing paediatric nursing diagnoses and inserting them into a case base in order to assess the effectiveness of the prototype in handling these cases in a structure conducive to retrieval, adaptation, indexing, and case comparison. This work presents as a result a computational tool for the health area, employing one of the artificial intelligence techniques, case-based reasoning (CBR). The small governmental nursing education institution in Bangladesh used in this study did not yet have the systemization of nursing care (NCS) and computerized support scales.

## 1. Introduction

Artificial intelligence (AI) offers techniques such as case-based reasoning (CBR) and fuzzy logic to develop knowledge-based systems that need to apply intelligence to provide solutions [1], and hence AI is defined as the constellation of elements (algorithms, robotics, and neural networks) that give software the possibility of being intelligent like human beings, that is, capable of learning through the database with little human interference [2]. Regarding AI techniques to help developers in the programming process, the requirement specifications should be described with the idea of finding an existing program that has the same specifications and then making the necessary changes, that is, making use of CBR in software engineering. Since its inception in the United States, case-based reasoning has grown rapidly in recent years. What began as a specialized area of inquiry has grown into a topic of broad interest, multidisciplinary research, and significant commercial potential. Case-based reasoning is just another problem-solving paradigm, but it is the contrast between it and the other artificial intelligence methodologies that distinguishes it. This paradigm is able to apply specific information from previous experiences, that is, concrete problem scenarios, rather than depending exclusively on broad knowledge of the problem area or establishing linkages along relationships between problem descriptions and conclusions. It is understood that the use of nursing care of systematization (NCS) requires nurses to master several skills [3, 4], and it is essential to follow theoretical support to better guide decision making, which in turn should be shared, whenever possible, with the patient [5, 6]. In this way, it is known that the NCS collaborates to provide safe, logical, and effective nursing care. The applicability of these records or technology in various clinical health situations, in which observations about the care needs of patients accompany the decision-making process about the care provided, helps in the subsequent evaluation of the results that are obtained with professional intervention. There is also the premise of organizing the management of nursing care, contributing to nurses' decision making, in order to guarantee patient safety at different levels of care. The goal of this project is to investigate and develop case-based reasoning for systematization of nursing care, bringing the state of the art in artificial intelligence to case-based reasoning and its application in the systematization of nursing care. To test the model, it was suggested that a diagnostic search prototype program be developed utilising case-based reasoning, an artificial intelligence technique [7, 8]. This prototype aided nurses in making proper diagnoses for possible solutions to the problems they were presented with, assisting them in their decision making and clinical judgement. Given the above, the present work is outlined such that the development and validation of an application (software) will raise the levels of knowledge of nurses and undergraduate students about NCS and its associated knowledge, in the context of nursing care.

Another aspect is the interplay between the stages of systematization of nursing care and the interventions required to restore patient health.

## 2. Methodology

The RBC artificial intelligence technique was used to translate real cases raised by nurses into the machine.Thus, it allows the integration between diagnoses, interventions, and nursing results according to the need suggested by Sanson et al. [9, 10]. It includes a friendly interface with representation of models of the human body in three dimensions, very close to the real one, facilitating the acquisition of physiological, biological, psychological, and social data. The first step to implement the proposed architecture presented in the previous section as in Figure 1 using case-based reasoning is to carry out a preliminary evaluation of the experiences. The second step is the definition of attributes for the representation to formulate “form like.” The third step is to define the case retrieval methods. The fourth step proposes a flexible interface for data acquisition which will be responsible for sending the characteristics necessary to perform the case search in the base.

### 2.1. Representation of Cases

To represent the cases, it is necessary to define the descriptors that describe the case that contemplates the problem, the solution, and the results or other information pertinent to the application domain. Furthermore, the descriptors can be used as indexes for retrieving the base cases and can lead to the adaptation of the solution of a case depending on the applied context. To find the cases relevant to a given problem, it is necessary to use attributes considered relevant to the case that promote the differentiation between one case and another, similar to the indexes of books that use key terms to help in finding the desired subject. The definition of useful attributes is a difficult task. In the extraction of attribute values in the functional approach used, even the extracted descriptors cannot always be used as an index, in the context of nursing a good example that can be given is the name of the diagnosis. Although it is important for the user, this does not mean that it can be used as an index because the problems found lead to the main objective, the diagnostic inference, or, in other words, the nursing diagnosis. Descriptors can be defined by an expert in the domain, as it determines the solutions to a problem that requires a domain of knowledge. It works in tandem with the books Nursing Outcomes Classification (NOC) and Nursing Interventions Classification (NIC), which describe the expected outcomes and the interventions required to achieve those outcomes.

### 2.2. Retrieval of Cases

The purpose of the case retrieval phase is to find cases or a set of cases that contain a useful solution for the current situation. To perform this recovery in order to perform this comparison, it is necessary to combine the description of the current problem with the existing situation in the knowledge base, which is composed of several previous experiences. It is necessary to use similarity functions that can be global or local depending on the application domain. A similarity list is created by comparing each case's characteristics to those of others in the database. If the search for identical cases did not yield any results, the list can be used to identify similar cases that can be used to adapt to a given situation. Using global similarity already compares the input cases' attributes to the characteristics of cases already stored in the case bank, and this comparison is done using a global similarity metric as described in equation (1) [11, 12], where *N* denotes the new case, *C* represents a case in the case bank's memory and has *I* attributes, *f* denotes the similarity function that compares attribute 1 of the new case *N* to the base case *C*, and *W*  is the degree of importance. When looking for similar examples, Figure 2 shows how this is performed.

(1) $$\begin{array}{c} \text{Sim}\left(N,C\right)=\int_{i=1}^{n}f\left(Ni,Ci\right)\times Wi. \end{array}$$

The operation of the diagnostics researcher (DR) consists of obtaining the data that correspond to the signs and symptoms sent by the data acquisition interface.

### 2.3. Interface for Data Acquisition

The Freemind 2 program may be used to build a customizable XML form for the information acquisition interface, which displays the inspired information in the human mental model by linking ideas and facts to various media (files), images, sounds, movies, and so on, also known as a conceptual map (Figure 3). Nurses can quickly and easily construct their own forms using this tool, and it can even be done by the nurse himself. In addition, it is possible to connect the tool's fields in three dimensions to human anatomy. An XML file, shown in Figure 4, will be the end product of this procedure, and it will be used by the system that creates the user interface. Simply changing the mental map and the case base to the new paradigm [13] will make this interface more adaptable to various nursing specialties as well as other health-related contexts. It will be possible to develop nursing forms with greater agility and speed than with traditional programming approaches, ensuring that information is always up-to-date and that users do not have to wait months for a new version of software that adapts their interface to the latest reality. These techniques can also be applied to the construction of data acquisition interfaces for Java-enabled mobile devices. Figure 4 depicts a three-dimensional human body with two primary goals: first, to make data collection easier, and second, to serve as a tool for teaching physiological, biological, and emotional phenomena to patients, in order to make the human body's representation more real and pleasant than traditional methods, which contain hundreds of clinical terms that must be interpreted and understood. Additional media can be included, such as sounds, photographs, and videos related with the desired event, allowing for a better understanding of the processes involved.

### 2.4. The Technologies Used to Implement the Tests

The main technologies used in the development of the prototype for the automation of nursing processes are as follows: Java Micro Edition (JavaME); Java Development Kit (JDK 1.6.0); Java Platform Micro Edition Software Development Kit; Eclipse (3.x); JColibri; Blender 3D; Mobile 3D Graphics API (M3G); and eXtensible Markup Language (XML).

## 3. Implementation and Results

In order to evaluate and approve the proposed system, the implementation of the prototype software was carried out following the Brazilian and international standards (ISO/IEC) which deals with software quality and system ergonomics. In this section, the cited standards that guided the elaboration of the questionnaire used to evaluate the proposal of this system are presented.

### 3.1. Interface for Data Acquisition

As shown in Figure 4, this model portrays a twelve-year-old child with some of the indications and symptoms that the nurse might find during exams. As a consequence of this project, the interface test using a three-dimensional (3D) human body in a Java environment was implemented and executed. One goal of this interface is to make it easier to collect data, and another is to help patients better understand their physiological, biological, and emotional states by providing a more realistic and intuitive visual representation than the traditional methods, which may contain hundreds of clinical terms that must be interpreted and comprehended. Aside from adding images and sounds associated with the desired event for a better understanding of the phenomena involved, it is also possible to record deformations in the three-dimensional model injuries as a result of some pathology or some medication side effects, such as stains, bruises, skin lesions, and so on.

It was important to design a program that could extract data from the Freemind form made by the user in order to propose a flexible interface that combines with the three-dimensional model. This is why a program called “interface generator,” which can link form fields to 3D models generated by Freemind, has been developed to read the XML files generated by Freemind and provide the results in a certain structure. Making use of the three-dimensional object modeller MakeHuman [14], the source code can replicate and even deform human traits like age, weight, height, and sex. This adds a high degree of realistic realism.

### 3.2. Simulation in a Mobile Environment

As soon as Blender 3D's m3g file was exported, concepts for reading these files on cell phones were applied [13]. The Java Platform Micro Edition Software Development Kit 3.0 results in a three-dimensional representation of the human body on the cell phone screen.

### 3.3. Diagnostic Researcher

A framework known as “JColibri” was utilised to create the diagnostic researcher (DR), which provides procedures for retrieving, reusing, reviewing, and retaining cases such as the Tex-current CBR application. For the development of RBC applications, this framework provides detailed documentation and models as well as a smaller learning curve than other frameworks. The JColibri Textual CBR module served as the foundation for the diagnostic search engine. An initial case base with 17 nursing diagnoses (cases) taken from the NANDA book was needed for this step. The case base was formatted according to the framework's specifications. There are highlighted and annotated sections of the DR. By using the “List Cases” window to display all diagnoses contained in the case database, including internationalisation techniques that allow multiple nurses to use the system from different countries and regions, for those who want to find nursing diagnoses quickly, they can use a diagnostic search engine that does inference to the diagnosis by entering defining characteristics of nursing diagnoses. Integration of DR and 3D interface was next, offering a more comfortable and realistic environment for nurses, allowing for more agility in data collecting and diagnostic inference, resulting in a good response from nurses.

### 3.4. Experimental Evaluation of OpenRBCenf

With the objective of promoting the health and safety of computer users, ensuring that they operate the equipment with maximum efficiency and comfort, BNC was created, which considers the point of view of the user in aspects such as usage and performance, demonstrating satisfaction with the interaction between the user and the system. The BNC standard divides the usability evaluation into three parameters: effectiveness—the measure is performed by the percentage of tasks performed correctly versus the total number of tasks that will be performed; efficiency—the measure considers the relationship between efficiency and the total time spent by the user to complete the task; and satisfaction—it refers to the identification of how certain tasks are performed by the user in a certain context of use. The requirements and recommendations related to software, hardware, and the environment involved with usability are defined in Bangladesh Nursing Council (BNC). The described standards point to which characteristics could be evaluated in the OpenRBCenf described in this section. For the evaluation of OpenRBCenf, the standard questionnaire adopted from Butt et al. [16] was used. The same questionnaire was applied to nursing students and nurses specialized in paediatric oncology at the Khulna Govt. Nursing Institute, Khulna, Bangladesh. In addition to objective questions with scores ranging from 1 to 5, being very dissatisfied to very satisfied, respectively, evaluating the level of satisfaction of each item questioned, there were also direct objective questions such as sex and whether or not he had already used software that uses third-dimensional interaction graphics technology, very common in games. Even the evaluator could give suggestions about improvements contributing to the improvement of the project and finally the expectation created by the software.

### 3.5. Opinion Survey Evaluation Result

OpenRBCenf was evaluated using two distinct samples: a group of nursing students in their final year of study and a group of paediatric oncology nurses. The results are shown graphically in Figures 5–13. There were two main goals for the presentation: first, to see if the system could be used by future nurses with little experience, and second, to see whether the technology could be utilised to educate and learn nursing ideas.

## 4. Conclusions and Suggestions

### 4.1. Conclusion

In conclusion, this article describes the proposal of an application to assist nursing professionals in their daily practice, and it is expected that its use will aid in the promotion of nursing diagnoses derived from patients' vital signs, other data, and the professional nurse's clinical and critical care judgement. It is important to emphasize that the possible use of this type of technology reaffirms the nursing practice regarding the use of a tool that allows the individualization of care, transforming the practice and serving as a basis for interventions, introducing the scientific method, with the objective of identifying existing problems and allowing the professional to make faster and more efficient decisions. The items covered in this standard made it possible to design a questionnaire for the acquisition of important data. When nurses' experiences were documented in the form of cases, it became possible to compile a large amount of data that can help nurses make new discoveries about nursing diagnosis and improve their procedures by analysing previously solved case studies. With this validation, the program may be expanded to other medical areas and/or specializations, since it has a framework that allows for the required changes to adapt to new demands. These aspects point to the necessity to continue implementing the system's subsequent stages in order to provide health professionals with a comprehensive and efficient working tool.

### 4.2. Suggested Future Works

One of the objectives is to find a storage structure that can improve the outcomes. One option is to use the archetype model, which allows storing and relating clinical notions. Taking measures of blood pressure, heart rate, pulse, body temperature, etc. can be described in terms that complement their meaning, such as which gadget will be used to measure heart rate or body temperature. The stethoscope is used to measure the patient's heart rate and the thermometer to assess their body temperature, thus storing the knowledge required to execute a task. Opener employs this storage structure for clinical ideas. The interaction between the stages of systematization of nursing care and the interventions that nurses must perform to restore the patient's health is another phase

## Figures and Tables

**Figure 1:** Proposed architecture of the project.

**Figure 2:** OpenRBCenf working architecture.

**Figure 3:** The paediatric nursing assistance systematization form using Freemind.

**Figure 4:** Physical examination using the human body in 3D.

**Figure 5:** Opinion survey evaluation result for the question: have you ever used software that uses three-dimensional interaction?

**Figure 6:** Opinion survey evaluation result for the question: what did you think of the experience? (Acceptability of the proposed interface).

**Figure 7:** Accuracy evaluation. (a) Grades given to software accuracy (by groups of evaluators). (b) Overall accuracy assessment.

**Figure 8:** Maturity assessment. (a) Grades given to software maturity (by groups of evaluators). (b) General assessment of maturity.

**Figure 9:** Assessment of intelligibility. (a) Grades given to software intelligibility (by groups of evaluators). (b) General assessment of intelligibility.

**Figure 10:** Evaluation of software efficiency in relation to time. (a) Grades given to the apprehensibility of the software (by groups of evaluators). (b) General apprehensibility assessment.

**Figure 11:** Evaluation of operability. (a) Grades given to the operability of the software (by groups of evaluators). (b) Evaluation of operability.

**Figure 12:** Evaluation of software efficiency in relation to time. (a) Grades given to efficiency. (b) Efficiency with respect to time.

**Figure 13:** Grades assigned to all items (general system assessment).

## Data Availability

The data used to support the findings of this study are included within the article.
